RETRACTED

# Efficacy of the Panax Notoginseng Ejiao Suppository in the Treatment of Patients with Ulcerative Proctitis and Its Effect on Inflammatory Response and Immune Function

**DOI:** 10.1155/2022/1479964

**Published:** 2022-09-21

**Authors:** Yu Liu, Yingjie Sun, Xince Wang, Dongsheng Wang, Li Zeng, Qingge Lu

**Affiliations:** Department of Anorectal, Tangshan Traditional Chinese Medicine Hospital, No. 3 Kangzhuang Road, Lubei District, Tangshan City, Hebei Province, China

## Abstract

**Objective:**

To investigate the efficacy of the Panax notoginseng Ejiao suppository in patients with ulcerative proctitis and its effect on inflammatory response and immune function.

**Methods:**

This study recruited 100 patients with ulcerative proctitis who were hospitalized to our hospital's anorectal outpatient department between May 2015 and October 2020. They were randomly separated into either a control or a study group, with 50 cases in each. The control group received the mesalazine suppository, whereas the study group received the Panax notoginseng Ejiao suppository. Outcome measures included clinical effectiveness, inflammatory response, and immunological state of patients.

**Results:**

The total efficiency in the study group was significantly higher than that in the control group (*P* = 0.019). The Mayo score and Baron endoscopic score between the two groups were significantly decreased after treatment, with lower results in the study group (*P* < 0.05). The inflammatory variables were dramatically reduced following therapy, with the study group doing worse. Following treatment, the number of Th 17 cells declined dramatically in both groups, while the proportion of Treg cells increased significantly, with greater alterations of Th17 cells and Treg cells observed in the study group than those in the control group (*P* < 0.05). The Panax notoginseng Ejiao suppository resulted in significantly shorter time lapses before symptom alleviation and a lower incidence of recurrence at 6 months after treatment versus mesalazine suppository (*P* < 0.05).

**Conclusion:**

In patients with ulcerative proctitis, the Panax notoginseng Ejiao suppository significantly improves clinical efficacy, reduces the incidence of recurrence, mitigates inflammatory response, and improves immune function.

## 1. Introduction

Ulcerative colitis is an idiopathic and chronic inflammatory disease of the colorectal mucosa, and approximately 30% of cases with inflammation involve only the rectum, which is termed ulcerative proctitis [1]. Patients with ulcerative proctitis have rectal bleeding, urgency, and tenesmus, and endoscopy can only reveal only diffuse rectum inflammation [2]. A prior study found that 28 percent of ulcerative proctitis cases had proximal dilatation, which proceeded to left-sided or pancolitis during five years [3].

RETRACTED

Currently, Western medicine management mostly involves hormones and immunosuppressive therapy. Intravenous steroid hormones are the preferred choice for severe UC, while hormone resistance has been reported in around 30% of patients, which is termed hormone-resistant UC [4]. Treatment alternatives are scarce for severe UC, especially for hormone-resistant UC, resulting in an increased risk of colonic resection [5]. Mesalazine is usually adopted as an initial treatment. Furthermore, topical mesalamine is preferable over topical steroids or oral mesalamine because suppositories are more effective than either topical or oral treatment alone in delivering the medicine to the rectum [6].

At present, the pathological mechanism of ulcerative proctitis is still unclear, and there are links to genetic, inflammatory, and autoimmune factors [7]. With the deepening of the research on the mechanism of ulcerative proctitis, the role of immune factors and inflammatory factors has been gradually investigated [8]. In traditional Chinese medicine (TCM), ulcerative colitis belongs to the category of “diarrhea” and “dysentery” and is predominantly attributed to lack of congenital endowment, weak spleen and stomach, or improper diet, or exogenous epidemic pathogenic poison, or emotional depression [9]. Traditional Chinese remedies such as Panax notoginseng and Ejiao are commonly used in ulcerative proctitis. Ejiao nourishes blood and moistens the lungs. Panax notoginseng increases blood circulation and alleviates blood stasis, dissolves rot, and reduces pain. Panax notoginseng and Ejiao have been shown in modern pharmacology to improve inflammatory factors and immunological function [10]. The Notoginseng Ejiao suppository is a new TCM preparation developed by our hospital that delivers the drug directly to the lesion site, nourishes blood, and promotes blood circulation, thereby enhancing long-term efficacy and reducing the incidence of recurrence. To this end, this study aimed at investigating the efficacy of the Panax notoginseng and Ejiao suppository in patients with ulcerative proctitis and its effect on inflammatory response and immune function.

## 2. Materials and Methods

### 2.1. Study Design

This study is an exploratory study, using a prospective randomized control design to explore the effect of the Panax notoginseng Ejiao suppository plus mesalazine suppository for the management of ulcerative proctitis. This study included 100 patients with ulcerative proctitis who were admitted to our hospital's anorectal outpatient clinic from May 2015 to October 2020. They were divided into a control group and a research group according to the ratio of 1 : 1 by the random method, with 50 patients in each group.

RETRACTED

The randomization was carried out using an online web-based randomization tool (freely available at http://www.randomizer.org/). For concealment of allocation, the randomization procedure and assignment were managed by an independent research assistant who was not involved in screening or evaluation of the participants.

The original sample size calculation estimated that 100 patients in each group would be needed to detect a 3-point difference between groups in a 2-sided significance test with a power of 0.8 and an alpha error level of 0.05.

The trial was done in accordance with the standards of Good Clinical Practice and the Declaration of Helsinki. The trial protocol and all amendments were approved by the appropriate ethics body at each participating institution. All patients provided written informed consent before enrolment. The trial protocol has been published online and is available with the full text of this article (Ethics No. HebTS178).

### 2.2. Inclusion and Exclusion Criteria

#### 2.2.1. Inclusion Criteria

The inclusion criteria were as follows: (1) patients with ulcerative proctitis diagnosed by gastrointestinal endoscopy and clinical symptoms; (2) patients aged 18–75 years, regardless of sex; (3) with mild-to-moderate active ulcerative proctitis, and the lesion is far from the anal verge within 15 cm; (4) with UC determined in an active stage by colonoscopy, sigmoidoscopy, and histopathological examination; (5) patients voluntarily signed the informed consent

#### 2.2.2. Exclusion Criteria

The exclusion criteria were as follows: (1) with Crohn's disease or other rectal diseases; (2) with a history of gastrointestinal surgery; (3) with severe heart, liver, kidney failure, myocardial infarction, acute stroke, and other underlying diseases; (4) with allergies to the drug in the study; (5) women who are pregnant or breastfeeding.

### 2.3. Treatment Methods

#### 2.3.1. Control Group

The control group was treated with 0.25–0.5 g of the mesalazine suppository (Vifor AG Zweigniederlassung Medichemie Ettingen, approval number: H20100126), thrice daily after defecation. The suppository was inserted into the anus with a hygienic finger cot until reaching the position where the resistance easily disappeared. The duration of treatment was 8 weeks.

#### 2.3.2. Study Group

The study group was treated with the Panax notoginseng Ejiao suppository on the basis of the control group. The preparation method of the Panax notoginseng Ejiao suppository was as follows: Panax notoginseng and Ejiao were crushed into fine powders, the rest of the medicines were decocted with water twice, and the decoction juice was mixed, filtered, and filtrated to a thick paste, which was mixed with the fine powder, dried, stirred evenly, and injected into a plug to mold into a suppository. The specific drugs are as follows: Panax notoginseng, Ejiao, Treats, Burnet, Lithospermum, Poppy Shell, Sophora flavescens, Rhizoma Bletillae, Pulsatilla, Coptidis, Ash Bark, and Rhizoma Corydalis, whose drug ratio is 3 : 3 : 10 : 10 : 10 : 6: 6 : 6 : 10 : 10 : 10:10. The duration of treatment was 8 weeks.

RETRACTED

### 2.4. Outcomes

#### 2.4.1. Disease Activity

After 8 weeks of treatment, the Mayo scale [11] was used to evaluate the disease activity. The Mayo score included the number of defecation, blood in the stool, endoscopic findings, and the physician's overall evaluation. It was scored from 0 to 12, with higher scores representing more severe symptoms.

#### 2.4.2. Condition of Rectal Mucosa

After 8 weeks of treatment, the Baron endoscopic score [12] of the two groups of patients was recorded to evaluate the condition of rectal mucosa, with 0 for colonic mucosa without congestion, 1 for mucosal congestion but no bleeding, 2 for obvious mucosal congestion that was granular, brittle, and easy to bleed, and 3 for mucosal ulcer and spontaneous bleeding.

#### 2.4.3. Clinical Efficacy

After 8 weeks of treatment, the clinical efficacy was evaluated according to the frequency of defecation and rectal mucosa, and it was divided into cured, markedly effective, effective, and ineffective.

Cured was defined as follows: the frequency of defecation is normal, there is no blood in the stool, and the rectal mucosa under the endoscope is normal. Markedly effective was defined as follows: the frequency of defecation is increased by 1–2 times/day compared with the normal frequency, and the frequency of blood in the stool is less than half of the frequency of defecation, with rectal mucosal erythema, reduced vascular texture, and mild brittleness under endoscopy. Effective was defined as follows: the frequency of defecation is increased by 3–4/day compared with the normal frequency, most of the time the blood was mixed in the stool, and the rectal mucosa under endoscopy is obviously erythema, lack of vascular texture, brittleness, and erosion. Ineffective was defined as follows: the frequency of defecation is increased by 5 times/day compared with the normal frequency or more, persistent bleeding, spontaneous bleeding of the rectal mucosa under endoscopy, and ulceration.

#### 2.4.4. Inflammatory Factors and Immune Function

After 8 weeks of treatment, fasting venous blood was collected from patients; ELISA was used to determine the concentrations of nuclear factor kappa-B (NF-*κ*B), tumor necrosis factor (TNF)-*α*, and interleukin (IL)-8; flow cytometry was used to determine the ratio of Th17 and Treg cells; and the ratio of Th17/Treg was calculated.

RETRACTED

#### 2.4.5. Follow-Up Outcomes

All patients were followed up for 6 months after operation, and the recurrence was recorded.

### 2.5. Statistical Analysis

The normality of the sample was determined with the Shapiro–Wilk test. Descriptive statistical data were evaluated with the exploratory analyses of the Tukey test. Quantitative mean data (PES/WES, ISQ, and B.L.) were assessed with the nonparametric Wilcoxon–Mann–Whitney *U* test to analyze the inferential statistics.

SPSS 22.0 software was used for data sorting and statistical analysis. Measurement data and enumeration data were expressed as mean ± standard deviation and rate, respectively, and *t* test and chi-square test were used to compare whether there were statistical differences between groups. Relapse-free survival time was assessed by Kaplan–Meier. *P* < 0.05 was regarded as a statistically significant difference.

## 3. Results

### 3.1. Baseline Characteristics

The patient characteristics between the two groups were comparable (*P* > 0.05) (Table 1).

### 3.2. Clinical Efficacy

The clinical efficacy of the two groups was compared after 8 weeks of therapy. 30 cases were cured in the control group, 5 cases were markedly effective, 4 cases were effective, and 11 cases were ineffective, for a total effective rate of 78.00% (31/42); 42 cases were cured in the study group, 5 cases were markedly effective, 2 cases were effective, and 3 cases were ineffective, for a total effective rate of 94.00% (47/50). The total effective rate in the study group was significantly higher than that in the control group (*P* = 0.019) (Table 2).

### 3.3. Mayo Score and Baron Endoscopy Score

There was no significant difference in the Mayo score and Baron endoscopic score between the two groups before treatment (*P* > 0.05), and the parameters were significantly decreased after treatment, with lower results in the study group (*P* < 0.05) (Table 3).

### 3.4. Inflammatory Factor Levels

The inflammatory factors were similar the two groups before treatment (*P* > 0.05), and the indices were significantly decreased after treatment, with lower results in the study group (*P* < 0.05) (Figure 1).

### 3.5. Immune Indices

Before treatment, the proportion of Th 17 and Treg cells did not differ between the two groups (*P* > 0.05). After treatment, the proportion of Th 17 in the two groups decreased significantly, while the proportion of Treg cells increased significantly, and the decrease and increase in the study group were more remarkable than those in the control group (*P* < 0.05) (Table 4).

RETRACTED

### 3.6. Time Lapses before Symptom Alleviation

The Panax notoginseng Ejiao suppository resulted in significantly shorter time-lapses before symptom alleviation versus mesalazine suppository (*P* <0.05) (Table 5).

### 3.7. Follow-Up Results

The recurrence of patients was monitored after therapy. In the control group, there were 6 cases of recurrence at 3 months and 15 cases at 6 months following treatment; in the study group, there were 2 cases at 3 months and 5 cases at 6 months. At 3 months following treatment, there was no significant difference in the incidence of recurrence between the two groups (*P* > 0.05). The recurrence rate at 6 months after treatment in the study group was significantly lower than that in the control group (*P* < 0.05) (Table 6).

## 4. Discussion

UC is a chronic idiopathic inflammatory bowel disease of the mucosa of the colon and rectum, with varying degrees of inflammation of the mucosa from the rectum to the proximal colon. UC predominates in adults aged 30 to 45 years and presents with abdominal pain, diarrhea, dyspepsia with food pressure, nausea, and vomiting. The pathogenesis of UC has not been fully determined and is associated with genetic susceptibility, epithelial barrier defects, and dysregulated immune response [13]. The etiology of ulcerative proctitis remains poorly understood, and it is closely related to the host response caused by foreign substances, genes, and immunity [14]. The disease occurs mostly in young adults, and no complete cure is available. Western medical treatment is based on aminosalicylic acid preparations, glucocorticoid antibiotics, and immunosuppressive drugs, which provide symptom relief of ulcerative colitis. Sulfasalazine is the main treatment drug, including Edissa and mesalazine. Corticosteroids, prednisone, or dexamethasone can significantly alleviate symptoms during acute exacerbations, but long-term use of corticosteroids is associated with disease relapses [15].

About 20% to 30% of patients with severe ulcerative proctitis are eventually converted from conservative treatment to surgical management [16]. The most common therapy for ulcerative proctitis is topical mesalazine. Inflammatory bowel tissue from individuals with inflammatory bowel illness enhanced leukocyte migration and increased the synthesis of aberrant cytokines and arachidonic acid metabolites, including leukotriene B4 and free radicals. Mesalazine blocks leukocyte chemotaxis, diminishes cytokine and leukotriene synthesis, and scavenges free radicals. The mesalazine suppository works directly on inflammatory intestinal tissue and has no pharmacological effects via absorption [17]. UC belongs to the category of “prolonged dysentery” in TCM. Weak spleen qi is the basis of the disease, and external evil, poor diet and emotional disorders are the main triggers. The onset of the disease is related to the large intestine and the dysfunction of the spleen, liver, kidney, lung, and other organs. The disease is usually caused by poor diet; fatty, sweet, and thick taste or abnormal innate endowment; emotional and mental disorders; and excessive labor and fatigue, resulting in injury to the spleen and stomach, stagnation of dampness and heat in the large intestine, and blood and qi fighting against each other and stagnation of qi and blood, resulting in injury to blood channels [18].

RETRACTED

In this study, the Panax notoginseng Ejiao suppository significantly potentiates the clinical efficacy, shortens the time lapse before symptom relief, reduces the magnitude of disease activity, improves the state of rectal mucosa, and lowers the long-term recurrence incidence. Previous research has shown that TCM is beneficial in ulcerative proctitis. In TCM, the disease is promoted by wet steaming and heat, qi, and blood coagulation, according to the local syndrome differentiation of ulcerative proctitis [19]. The Notoginseng Ejiao suppository prepared by our hospital offers the benefits of TCM retention enema with simple use and high efficiency. Several studies have shown that Panax notoginseng reduces mucosal damage and promotes mucosal repair. In a rat model of colitis induced by sodium dextran sulfate, the use of Panax notoginseng ethanol extract promotes the repair of colonic mucosa and microvascular damage in rats with colitis, reduces the inflammatory response, and lowers the disease activity scores [20]. In addition, in a colitis rat model, Panax notoginseng extract upregulates the expression of ATP4a in mitochondria in colonic mucosal epithelial cells to improve glycolysis, which is strongly associated with the activation of mitochondrial aerobic oxidation [21].

The results of the present study indicate that the Panax notoginseng Ejiao suppository for ulcerative proctitis effectively alleviated clinical symptoms, controlled inflammation, promoted ulcer healing, and improved patients' quality of life. The reasons for this analysis may be that (1) the Panax notoginseng and Ejiao suppository formula contains Panax notoginseng with the effect of stopping bleeding and nourishing blood, activating blood circulation, and removing blood stasis, and Ejiao with the effect of stopping bleeding and nourishing blood [22]. In addition, as a pure traditional Chinese medicine preparation refined from the natural insect herb American cockroach, the active ingredients of Kangfu Xinye contain polyols, peptides, and mucosylate, which have the effects of acid suppression, anti-inflammation, improvement of microcirculation in mucosal wounds, promotion of granulation tissue proliferation, and acceleration of repair and regeneration of diseased tissues [23]. (2) This study used rectal local drug delivery, which allowed the drug to directly reach and act on the ulcer site, effectively prolonging the action time of the drug in the ulcer site and increasing the concentration of the drug in the ulcer site. (3) The present study on ulcerative proctitis effectively evaded the drawback of oral drugs in ulcerative proctitis which is difficult to achieve effective local drug concentrations [24].

RETRACTED

Experiments have shown that in inflammatory bowel disease, local CD4+ T cells infiltrate and show functional abnormalities. CD4+ T cells mainly consist of four subpopulations of Th1, Th2, Th17, and Treg cells [25]. Under normal conditions, Th17 and Treg are in dynamic balance in the body, thus maintaining the stability of the body's environment and their imbalance results in inflammation responses and diseases. During the development of UC, overexpression of Th17 cells and deficiency of Treg cells can lead to intestinal inflammation. Th17 cell differentiation is regulated by transforming growth factor-*β* (TGF-*β*)/interleukin-6 (IL-6) or IL-21 and requires the involvement of key transcription factors retinoic acid-related orphan receptors [26, 27]. The Th 17 cells and Treg cells are CD4+ T lymphocytes. Th 17 cells cause inflammatory damage by secreting pro-inflammatory cytokines, and Treg cells inhibit inflammatory damage by secreting anti-inflammatory cytokines. In the present study, the study group showed significantly lower inflammatory factors than the control group, indicating a better immune function in patients of the study group. Ejiao contains collagen, which can be decomposed in the body to obtain a variety of amino acids to enhance immunity. Research has shown that donkey-hide gelatin could enhance the immune system by targeting and increasing T cells in the spleen [28]. Additionally, it has been reported that donkey-hide gelatin inhibits the inflammatory response and adipocyte dysfunction in adipose tissue induced by intestinal microbial lipopolysaccharide [29, 30].

This study has the following limitations: the cases in this study came from the inpatients of the gastroenterology department of our hospital, with a single case source and small sample size, and the observation period was short. This subject failed to reflect the significance of classical theory in terms of observed indicators. In addition, this study lacks a more scientific basis because of the absence of animal testing. Future studies can further expand the source of cases and sample size, design indicators that reflect the significance of medicinal foods, and extend the observation period and follow-up so as to obtain more complete data and more significance of the study.

RETRACTED

## 5. Conclusion

In patients with ulcerative proctitis, the Panax notoginseng Ejiao suppository significantly improves the clinical efficacy, reduces the incidence of recurrence, mitigates inflammatory response, and improves immune function. In addition, the drug acts directly on the ulcer surface without passing through the stomach and intestines, avoiding the influence of digestive juices on the drug, reducing the first-pass effect of the liver, and improving bioavailability. It is also portable and easy to use, which fills the research gap and has effective effects and provides therapeutic benefits to the patients with ulcerative colitis.

## Figures and Tables

**Figure 1:** Comparison of inflammatory factor levels between the two groups; CRP, TNF-*α*, IL-6, and IL-8 indices were compared between the two groups before and after therapy to evaluate inflammatory factor levels. The results revealed that the inflammatory variables in the two groups were identical before treatment, and the indices were dramatically reduced after treatment, with the study group having lower values.∗∗ means *P* < 0.01, ∗∗∗ means *P* < 0.001.

**Table 1:** Baseline data.

	Study group (*n* = 50)	Control group (*n* = 50)	*t*/*χ*^2^	*P*
Age (year)	42.15 ± 11.25	44.65 ± 13.46	1.008	0.316
Gender			0.372	0.542
Male	28	31		
Female	22	19		
BMI (kg/m^2^)	25.19 ± 5.23	26.21 ± 5.18	0.980	0.330
Course of disease	4.59 ± 1.02	4.71 ± 1.13	0.557	0.579
Involved sites			0.679	0.410
Rectum	21	17		
Rectosigmoid colon	29	33		

**Table 2:** Comparison of clinical efficacy between the two groups of patients.

	Cured	Markedly effective	Effective	Ineffective	Total effectiveness
Control group (*n* = 50)	30	5	4	11	78.00%
Study group (*n* = 50)	42	5	2	3	94.00%
*χ* ^2^					5.316
*P*					0.021

**Table 3:** Comparison of modified Mayo score and Baron endoscopic score between two groups of patients ($\bar{x}\pm s$).

	Modified Mayo score		Baron endoscopic score	
	Before treatment	After treatment	Before treatment	After treatment
Control group (*n* = 50)	7.52 ± 1.12	3.25 ± 0.65	1.86 ± 0.37	0.72 ± 0.18
Study group (*n* = 50)	7.29 ± 1.43	2.79 ± 0.54	1.77 ± 0.32	0.48 ± 0.12
*t*	0.315	4.830	1.374	5.949
*P*	0.754	<0.001	0.173	<0.001

RETRACTED

**Table 4:** Comparison of immune indicators ($\bar{x}\pm s$, %).

	Th 17		Treg	
	Before treatment	After treatment	Before treatment	After treatment
Control group (*n* = 50)	18.25 ± 3.53	11.25 ± 2.85	4.02 ± 0.86	5.69 ± 1.16
Study group (*n* = 50)	17.19 ± 3.26	9.11 ± 2.26	3.95 ± 0.76	6.85 ± 1.42
*t*	1.560	4.160	0.431	4.473
*P*	0.122	<0.001	0.667	<0.001

**Table 5:** Comparison of symptom improvement time ($\bar{x}\pm s$, day).

	Stomach ache	Diarrhea	Mucous pus and bloody stool
Control group (*n* = 50)	5.36 ± 1.25	4.15 ± 0.95	7.28 ± 1.53
Study group (*n* = 50)	4.11 ± 1.13	3.26 ± 0.72	6.11 ± 1.26
*t*	5.245	5.280	4.174
*P*	<0.001	<0.001	<0.001

**Table 6:** Comparison of recurrences.

	3 months after treatment	6 months after treatment
Control group (*n* = 50)	6 (12.00%)	15 (30.00%)
Study group (*n* = 50)	2 (4.00%)	5 (10.00%)
*χ* ^2^	2.174	6.250
*P*	0.140	0.012
